The article "High-Resolution Microscopy to Learn the Nuclear Organization of the Living Yeast Cells" was retracted in 2024. Reasons: signs of a paper mill; suspected computer-generated content; unreliable results or conclusions; concerns about the data.

# High-Resolution Microscopy to Learn the Nuclear Organization of the Living Yeast Cells

**DOI:** 10.1155/2021/9951114

**Published:** 2021-08-27

**Authors:** Renjie Wang, Aiwen Huang, Yan Wang, Pengxin Mei, He Zhu, Qianqian Chen, Sankui Xu

**Affiliations:** College of Materials Science & Engineering, Henan University of Technology, Zhengzhou, China

## Abstract

The spatial organization of the nucleus is a key determinant in all genome activities. However, the accurate measurement of the nuclear organization is still technically challenging. Here, the technology NucQuant we created previously was utilized to detect the variation of the nuclear organization, including the heterogeneity of the nuclear geometry, the change of the NPC distribution along different cell cycle stages during interphase, and the organization of the nucleolus. The results confirmed that not only the growth rate and the NPC distribution are influenced by the carbon source; the nuclear shape is also impacted by the carbon source. The nuclei lost their spherical geometry gradually when the cell was cultured from the most to a less favorable carbon source. We also discovered that the nucleolus prefers to locate at the nuclear periphery, which was called the “genes poor region,” especially when the cells entered quiescence. Furthermore, the distribution of the NPC along the different stages during the interphase was analyzed. We proposed that with the growth of the cell, the nucleus would grow from the surface of the NE flanking the nucleolus firstly.

## 1. Introduction

Chromosome spatial organization plays a key role in transcriptional regulation, DNA repair, and replication [1]. In eukaryotic cells in interphase, the chromosomes are segregated away from the cytoplasm by the nuclear envelope (NE). How do chromosomes organize in the eukaryotic nucleus is still an open question. In budding yeast, NE remains closed during the entire cell cycle, including mitosis. Past researches have uncovered few structural features characterizing the budding yeast nucleus in interphase: the spindle pole body (SPB), centromeres (CEN), telomeres (TEL), and nucleolus. In interphase, the nucleolus is organized in a crescent-shaped structure adjacent to the NE and contains quasiexclusively genes coding ribosomal RNA (rDNA) present on the right arm of chromosome XII. The genome structure and the nucleolar organization are intimately connected owing to the efficiency of rDNA transcription that plays an important role in the nucleolar organization [2]. Diametrically opposed to the nucleolus, the SPB tethers the CEN during the entire cell cycle via microtubules to the centromere-bound kinetochore complex [3–6]. TEL are localized in clusters at the NE [7, 8]. Consequently, chromosome arms extend outwards from CEN to the nuclear periphery, defining a Rabl-like conformation [9, 10]. Nuclear pore complexes (NPCs) are embedded in the envelope to control the nucleocytoplasmic transport of molecules [11]. Besides, components of the NPCs have been proposed to play a key role in the chromatin organization [12]. The NPC components, Nups, are connected to the chromosomes and regulate the expression of certain genes [13–16]. Therefore, the distribution of the NPCs on NE and the nucleolus organization need to be precisely defined to accurately explore eukaryotic nuclear organization.

The nucleus in budding yeast in interphase is always described as a sphere of radius ~1 *μ*m. However, the nuclear shape and size *in vivo* are dynamic [17]. Along the cell cycle, the nucleus adopts different morphologies and sizes. In the G1/S phase (or interphase), the nucleus is often described as a sphere; this structure is clearly established when yeast is growing in rich medium containing glucose [18]. Differential interference contrast (DIC) microscopy research indicated that the nucleus is more or less spherical [19]. Transmission Electron Microscopy (TEM) analysis of ultrathin (60-80 nm) sections of an entire nucleus showed that the yeast nucleus in interphase undergoes a twofold increase in volume from G1 to S phase [20]. The “Nucloc” program created by Berger et al. to analyze the “genes territories” in the nucleus fits the NE through spherical simulation based on the detection of labeled NPCs; the results of this approach showed that the median budding yeast nucleus in interphase can be approximated as a sphere of ~1 *μ*m radius [17]. However, the approximation of the yeast nucleus as a sphere is oversimplified, the nuclear shape being dynamic along the cell cycle and in different conditions [21]. Additionally, due to the existence of the aberration along the *Z* axis, the spherical fitting of the nucleus in interphase is not precise [22].

Accurate determination of the nuclear organization using fluorescence microscopy is technically challenging [23, 24]. The fit of the NE position is still controversial because of the resolution barrier in fluorescent microscopy: 200 nm in *X*-*Y* and about 500 nm in *Z* axis [25]. In budding yeast, fluorescent-labeled NPCs appear as typical punctate rings staining the NE which can perfectly be used to reconstruct the NE structure in 3D [20, 23]. Here, we used “NucQuant,” an optimized automated image analysis algorithm we developed in our previous work [22], which can automatically localize fluorescently labeled NPCs and correct the detection bias resulting from optical spherical aberration along the *Z* axis to accurately compute an approximation of the NE in 3D. In addition, it also can detect the structure of the labeled nucleolus. This approach allowed us to precisely measure the heterogeneity of the nuclear shape and the NPC distribution along interphase. Based on this technology we could evaluate the nucleolus structure and organization in interphase. We also detected the change of the NPC distribution along the NE correlated with the cell cycle stage.

## 2. Materials and Methods

### 2.1. Yeast Strains

Genotypes of the strains used in this study are described in Table 1.

### 2.2. Fluorescence Microscopy of Living Yeast Cells

#### 2.2.1. Cell Culture

Yeast media were used as previously described [22]. The Yeast Extract Peptone Dextrose Medium (YPD) is made of 1% yeast extract, 2% peptone, and 2% dextrose. Synthetic complete media (SC) is made of 0.67% nitrogen base w/o amino acids (BD Difco, USA), 2% dextrose supplemented with amino acid mixture (AA mixture Bio101, USA), adenine, and uracil. Cells were grown overnight at 30°C in the Yeast Extract Peptone (YP) media containing 2% carbon source, cells were diluted at 10^6^ cells/mL in rich glucose, galactose, or raffinose containing media. Cells were harvested when OD600 reached 4 × 10^6^ cells/mL and rinsed twice with the corresponding SC media. Cells were spread on slides coated with corresponding SC patch containing 2% agar and 2% of corresponding carbon source. Cover slides were sealed with “VaLaP” (1/3 vaseline, 1/3 lanoline, and 1/3 paraffin). For short time starvation experiments, when OD600 reached 4 × 10^6^ cells/mL, cell culture was washed twice with YP media, resuspended at OD600 = 4 × 10^6^ cells/mL in YP (15%) media, and incubated for 2 hours at 30°C. For 7 days of progressive starvation experiments, we used YP containing 2% glucose media to culture the cells for 7 days.

#### 2.2.2. Confocal Microscope Image Acquisition

Confocal microscopy was performed as previously described [26]. Confocal microscopy was limited to 20 min after mounting and performed with an Andor Revolution Nipkow-disk confocal system installed on an Olympus IX-81, featuring a CSU22 confocal spinning disk unit (Yokogawa) and an EMCCD camera (DU 888, Andor). The system was controlled using the mode “Revolution FAST” of Andor Revolution IQ1 software (Andor). Images were acquired using an Olympus 100x objective (Plan APO, 1.4 NA, oil immersion). Single laser lines used for excitation were diode-pumped solid-state lasers (DPSSL) exciting GFP fluorescence at 488 nm (50 mW, Coherent) and mCherry fluorescence at 561 nm (50 mW, Cobolt Jive). A Semrock bibandpass emission filter (Em01-R488/568-15) allowed the collection of green and red fluorescence. Pixel size was 65 nm. For 3D analysis, Z-stacks of 41 images with a 250 nm Z-step were used. For microfluidic experiments, the fluorescence images can be acquired for more than 2 hours.

### 2.3. Image Analysis

Confocal images were processed and analyzed with a Matlab script NucQuant, the modified version of “Nucloc” combined with the correction of the aberration along the *Z* axis, which is available to download at GitHub (https://github.com/ogadal/nucquant). The nuclear shape was fitted by the 3D-NE model, and the cumulative distribution functions (CDF) of the sphericity of the NE were generated using the existing function in the NucQuant. The probability density distribution of detected NPCs along NE was generated using the existing function (Matlab). To calculate the position of the nucleolus relative to the NE, here, we modified the NucQuant algorithm about the detection of the nucleolus. All pixels of the nucleolus were detected and then corrected Z-aberration based on the NPC position of one perfect spherical nucleus. Schematical of NucQuant is presented in Figure S1.

## 3. Results and Discussion

### 3.1. Heterogeneity of the Nuclear Shape in the Cell Population

The cell nucleus is typically spheroidal or ellipsoid [17, 18]. However, the nuclear shape has high plasticity: in the same strain, the nuclei also have different shapes from cell to cell [27]. To study the heterogeneity of the nuclear shape in the interphase of one cell population, we utilized NucQuant to determine the NE with a 3D-NE model and measured the sphericity of each cell nucleus. Sphericity is one criterion to reflect how round an object is. The sphericity of a given object is the ratio between the surface area of a sphere which would have the same volume as that object to the surface area of the object [28]. For one perfect sphere, the sphericity index equals 1 and is maximal. A sphericity index lower than 1 indicates deviation from a perfect sphere. For one ellipsoid, the sphericity is ~0.92 when *a* : *b* : *c* = 1 : 1 : 2 (Figure 1(a)). The sphericity of the yeast nucleus was tested when the carbon source was changed from the most favorable to the less favorable carbon source. We confirmed that most of the nuclei in the interphase were close to spherical (the median sphericity is over 0.99). However, about 20% of the nuclei are rather ellipsoidal (sphericity below 0.95) (Figure 1(b); the samples are presented in Figure 1(d)). We also found that when the carbon source was changed to the less favorable carbon source ethanol, the sphericity clearly decreased compared with the favorable carbon source (Figure 1(b)). Consider the ~twofold reduction of the nuclear volume when changing from the most to a less favorable carbon source [22], we proposed that, when the carbon source changed from the most to a less favorable carbon source, the nuclear volume decreased anisotropic, which resulted in the nuclear shape tends to much more nonspherical. Actually, after the cells entered quiescence, ~70% nuclear lost their sphericity. So, we also explored the heterogeneity of the nuclear shape after the cells entered quiescence. The results clearly showed that after 7 days of starvation, most of the nuclei lost their sphericity (Figure 1(c)). We supposed that the nuclei will anisotropically shrink, which leads to most of the nuclei lost their spherical geometry, to control the limited consumption when the cells entered quiescence.

### 3.2. Heterogeneity of NPC Distribution in Different Interphase Stages

NPC probability density map reflects the distribution of the NPC clusters along the nuclear envelope (NE). In this research, to assess the NPC distribution along the interphase, we sorted nuclei in G1, S, and G2. During interphase, nuclear volume is continuously increasing, from G1 to G2 [29]. This property has an implication: the closer the cell is from the G1 stage, the smaller is the nucleus. Therefore, we sorted nuclei according to their volume: the small newborn G1 nuclei and the mother nuclei in the G1 phase, the middle nuclei in the late G1 phase and S phase, and the bigger nuclei in the late S phase and early G2 phase. The NPC distribution in small, middle, and big nuclei of cells grown on different carbon sources was analyzed with “NucQuant.” The results interestingly showed that the NPC distribution varied along the interphase stages, the NPCs gradually moved away from the NE flanking the nucleolus in interphase (Figure 2). In addition, it was also obvious that the NE elongated along the nucleolus direction with the cells growing.

The mechanism of the NPCs concentrated around the nucleolus for the small nuclei are still unclear. There is more and more evidence proving that in most mutants altering the nuclear shape, the NE preferentially elongates at the nucleolar side [30–33]. The nucleolus contacts extensively with the NE. NE flanking the nucleolus has very specific properties [32]. Previous research suggested that these specialized properties can prompt the transfer of the nucleolar materials to the cytoplasm without passing through the nucleoplasm [34]. We would prefer to link these properties to the cell cycle. After cell division, in the small nuclei, we can observe the NPCs are concentrated at the NE flanking the nucleolus. This might be a consequence of mitosis, with the hourglass shape and the nucleolus being the last nuclear domain to segregate. In the late G1, S, and G2 phases, the surface of the nucleus is increased from the NE flanking the nucleolus [35]. Thus, the NPCs at this site are gradually shifted away from the nucleolus. In addition, because of the increase of the nuclear surface, the distance between clustered NPCs increased which allows the localization microscopy to distinguish the close NPCs; this is also why we can detect more NPC from the big nuclei.

### 3.3. The Organization of the Nucleolus

The budding yeast has 100-200 ribosomal DNA (rDNA) units tandemly located on chromosome XII which is confined in the nucleolus. Only half of the rDNA copies are actively transcribed in *S. cerevisiae* [36]. Quantifying the intranuclear position of the nucleolus is essential for studying the spatial conformation of chromosomes. In budding yeast, the nucleolus contacts extensively with the nuclear envelope (NE) (Figure 3(a)). The research on the nuclear periphery, which was always seen as the silenced region, is significant to help us to understand the relation between chromosome organization and transcription activity. By using “NucQuant,” the peripheral location of the nucleolus in 3D could be accurately explored.

Our previous work has shown that the growth of cells was stopped and the nucleolar size decreased after the cells enter quiescence [22]. We were wondering if this change in the nucleolar size impacts its localization with respect to the nuclear periphery. To answer this question, we calculated the fraction of the nucleolus located at the nuclear periphery. We defined periphery as 1/3 of the nuclear volume uniformly distributed along the NE. The nucleolar periphery percentage is the proportion of the nucleolus at the nuclear periphery. It is clear that with such definition, the nucleolus was not restricted to the peripheral region: in asynchronous cells, we measured a median of ~60% of the nucleolus located at the nuclear periphery. After cells entered quiescence, the percentage of the nucleolus at the nuclear periphery is massively increased (Figure 3(b)). We proposed that the transcription of the rDNA was repressed; more rDNA units would be organized to the periphery region which caused the peripheral localization of the nucleolus, when the cells entered quiescence.

## 4. Conclusion

In this study, the heterogeneity of the nuclear organization, including the nuclear geometry, the distribution of the NPC along the NE, and the nucleolus organization, was successfully determined through the “NucQuant” technology. The nuclear would shrink anisotropically to control the limited consumption of the cell, which resulted in the nuclei lost their sphericity, when the carbon source changed from the most to a less favorable. Moreover, the NE increased from the surface of the NE flanking the nucleolus with the growing of the nuclear, which caused the variety of the NPC distribution along the NE close to the nucleolus. Furthermore, accompanying the shrink of the nucleus, the nucleolus also reorganized to the periphery region since the transcription of the rDNA was repressed.

## Figures and Tables

**Figure 1:** The heterogeneity of the nuclear shape in the cell population. (a) The sphericity of the perfect sphere (sphericity = 1) and the ellipsoid (sphericity = 0.92). (b) The change of the nuclear geometry in cell population cultured by different carbon sources, the sphericity of the nuclei decreases when the carbon source changed from the most favorable to the less favorable. (c) The distribution of the nuclear geometry after the cell population enters quiescence. (d) Two typical examples of the nucleus with different geometry *in vivo*, small blue spheres represent the detected NPC clusters.

**Figure 2:** The variety of the NPC distribution along the NE according to carbon sources. The NPC probability density maps based on analysis of asynchronous cells cultured with glucose (a), galactose (b), and raffinose (c). The small-sized nuclei are composed of the newborn nuclei and the mother nuclei in the G1 phase; the middle-sized nuclei consist of the nucleus in the later G1 phase and S phase. The nuclei in the later S phase and early G2 phase constitute the bigger-sized nuclei. The dashed yellow circle represents the nuclear envelope determined according to the “NucQuant” technology; the red curve represents the median nucleolus contour; the red small circle represents the median nucleolar centroid; *N* represents the number of the NPC clusters used to generate the cumulative percentage maps.

**Figure 3:** The change of the nucleolar organization after the cell population enters quiescence. (a) Schematic of the nucleus, nucleolus, and nuclear periphery region. Here, the periphery region was defined as the region that occupied 1/3 of the total nucleus at the periphery. The solid and dashed yellow circles represent the NE and the boundary of the nuclear periphery, respectively. (b) The reorganization of the nucleolus after the cell population enters quiescence, the nucleolus localized to the nuclear envelope closer.

**Table 1:** Genotypes of strain used in this study.

Name	Genotype
ycnod99-1a	*MATa His3-Δ1*, *leu2-Δ0*, *C*, *ura3-Δ0*, *ade2-801*, *lys2-801*, *lys2D::KAN-MX*, *nup49-Δ::HPH-MX6* + pASZ11-NupNop

## Data Availability

The data used to support the findings of this study are available from the corresponding author upon request.

## Supplementary Materials

Supplementary Materials Supplementary Figure S1 shows the schematic illustration of the “NucQuant” technology.
